The article "An Indole Alkaloid from a Tribal Folklore Inhibits Immediate Early Event in HSV-2 Infected Cells with Therapeutic Efficacy in Vaginally Infected Mice" was retracted in 2025. Reasons: errors in the methods; duplicated images; duplicated data; duplicate publication.

# An Indole Alkaloid from a Tribal Folklore Inhibits Immediate Early Event in HSV-2 Infected Cells with Therapeutic Efficacy in Vaginally Infected Mice

**DOI:** 10.1371/journal.pone.0077937

**Published:** 2013-10-22

**Authors:** Paromita Bag, Durbadal Ojha, Hemanta Mukherjee, Umesh Chandra Halder, Supriya Mondal, Nidhi S. Chandra, Suman Nandi, Ashoke Sharon, Mamta Chawla Sarkar, Sekhar Chakrabarti, Debprasad Chattopadhyay

**Affiliations:** 1 ICMR Virus Unit, ID and BG Hospital, Beliaghata, Kolkata, India; 2 National Institute of Cholera and Enteric Diseases, Beliaghata, Kolkata, India; 3 Department of Applied Chemistry, Birla Institute of Technology, Mesra, Ranchi, India; International Center for Genetic Engineering and Biotechnology, India

## Abstract

Herpes genitalis, caused by HSV-2, is an incurable genital ulcerative disease transmitted by sexual intercourse. The virus establishes life-long latency in sacral root ganglia and reported to have synergistic relationship with HIV-1 transmission. Till date no effective vaccine is available, while the existing therapy frequently yielded drug resistance, toxicity and treatment failure. Thus, there is a pressing need for non-nucleotide antiviral agent from traditional source. Based on ethnomedicinal use we have isolated a compound 7-methoxy-1-methyl-4,9-dihydro-3*H*-pyrido[3,4-*b*]indole (HM) from the traditional herb *Ophiorrhiza nicobarica* Balkr, and evaluated its efficacy on isolates of HSV-2 *in vitro* and *in vivo*. The cytotoxicity (CC_50_), effective concentrations (EC_50_) and the mode of action of HM was determined by MTT, plaque reduction, time-of-addition, immunofluorescence (IFA), Western blot, qRT-PCR, EMSA, supershift and co-immunoprecipitation assays; while the *in vivo* toxicity and efficacy was evaluated in BALB/c mice. The results revealed that HM possesses significant anti-HSV-2 activity with EC_50_ of 1.1-2.8 µg/ml, and selectivity index of >20. The time kinetics and IFA demonstrated that HM dose dependently inhibited 50-99% of HSV-2 infection at 1.5-5.0 µg/ml at 2-4 h post-infection. Further, HM was unable to inhibit viral attachment or penetration and had no synergistic interaction with acyclovir. Moreover, Western blot and qRT-PCR assays demonstrated that HM suppressed viral IE gene expression, while the EMSA and co-immunoprecipitation studies showed that HM interfered with the recruitment of LSD-1 by HCF-1. The *in vivo* studies revealed that HM at its virucidal concentration was nontoxic and reduced virus yield in the brain of HSV-2 infected mice in a concentration dependent manner, compared to vaginal tissues. Thus, our results suggest that HM can serve as a prototype to develop non-nucleotide antiviral lead targeting the viral IE transcription for the management of HSV-2 infections.

The article "An Indole Alkaloid from a Tribal Folklore Inhibits Immediate Early Event in HSV-2 Infected Cells with Therapeutic Efficacy in Vaginally Infected Mice" was retracted in 2025. Reasons: errors in the methods; duplicated images; duplicated data; duplicate publication.

## Introduction

Genital herpes is an incurable genital ulcerative disease, usually caused by herpes simplex virus type 2 (HSV-2), and represent one of the most serious public health concerns globally. The virus is transmitted during sexual intercourse and replicates in the genital epithelium, with life-long latency in dorsal ganglia [1]. More than 90% of genital herpes are caused by HSV-2 infections; which spread through unprotected sex, periodically reactivated and may cause fatal infections like acute encephalitis and meningitis in neonates and immune deficient patients [2]. It is reported that the immediate-early (IE) genes of HSV activate HIV-1 [3], Varicella-zoster virus [4] and human papillomavirus type 18 [5] genes, and is a significant risk factor for HIV/AIDS transmission [6]. Moreover, HSV‐2 can cross the placental barrier and affect foetus in early pregnancy, leading to spontaneous abortion or mental retardation of the foetus [7]. Furthermore, HSV-2 is known to transform infected cells into tumor cells [8] and have synergistic relationship with HIV disease progression [9]. Young women are biologically more vulnerable to genital infections than men to get these infections during vaginal intercourse [10]. A recent study showed that HSV-suppressive therapy can greatly reduce genital and plasma HIV-1 RNA load in co-infected patients [11], indicating that the risk of acquisition or transmission of HIV infection can be greatly decreased by reducing the spread of genital herpes.

Since 1974, HSV infections are managed with the nucleoside analogue acyclovir (ACV) which phosphorylated in the infected cells by viral *thymidine kinase* [12]. However, ACV fails to eradicate the virus from the infected cell or prevent recurrences, as it cannot counteract in the early stage of HSV infection [13]. Additionally, long term use of ACV or related drugs leads to the frequent development of drug resistant viruses, especially in immunocompromised individuals [16,17], implicating an increasing risk of HSV recurrence and treatment failure [18-20]. Moreover, till date no effective therapy [14] or vaccine [15] is available. Thus, new drugs with novel mode of action are required for the management and prevention of HSV infections. Here, we report the isolation of an antiviral compound from *Ophiorrhiza nicobarica* (International plant index Id: 758538-1), a traditional herb used by the Shompen and Nicobarese tribes of the Nicobar Islands, India, against skin ailments [21], having antimicrobial and antiinflammatory activities [22,23] with significant anti-HSV-2 activity. Further, we have demonstrated the *in vitro* mode of action and therapeutic efficacy of the isolated compound in Balb/C mice vaginally infected with HSV-2.

The article "An Indole Alkaloid from a Tribal Folklore Inhibits Immediate Early Event in HSV-2 Infected Cells with Therapeutic Efficacy in Vaginally Infected Mice" was retracted in 2025. Reasons: errors in the methods; duplicated images; duplicated data; duplicate publication.

## Materials and Methods

### Plant materials

*Ophiorrhiza nicobarica* Balkr. (Rubiaceae), a wild perennial herb, was collected from the Galathia River village, Great Nicobar Islands, India, in which no specific permissions were required as it was within the human habitat and not under any protected area. The herb, not under protected species, was identified by Dr. Sreekumar, Scientist, Botanical Survey of India (BSI), Andaman Nicobar Circle, Port Blair, and deposited in the Herbarium collection (Herbarium No. 9227) of the BSI, Port Blair, India. 

### Extraction, fractionation and identification of compound

Alcoholic extracts were prepared from the dried and coarsely powdered herb (100 g) with 1 L of MeOH (95%) for 48-72 h in a soxhlet extractor, collected, filtered and evaporated *in vacuo* to a residue at 40-45°C, with a yield of 7.8±0.2% (w/w). A part of the residue was stored in a dessicator for further study and the other part (32 g) was suspended in water and extracted with *n*-butanol, and then separately monitored by TLC. The *n*-butanol fraction (24 g) was subjected to Silica-gel CC, eluting with petroleum ether (PE), PE:CHCl_3_, CHCl_3_, and CHCl_3_:MeOH (at different ratios) and MeOH. The eluted fractions A (7 g), B (6 g) and C (8 g) were repeatedly subjected to Silica gel CC and monitored by TLC. Fraction A was positive for terpenoid, fraction B to phytosterol and fraction C for alkaloid. All fractions were separately isolated and subjected to CC by aluminium oxide eluted with PE, PE:CHCl_3_, CHCl_3_, and CHCl_3_:MeOH (at different ratios) on TLC. Fractions A and B were combined, condensed, recrystallized and identified by IR, NMR and mass spectroscopy [24]. The ^1^H and ^13^C NMR spectra recorded at 600 and 150 MHz in a Bruker AVANCE600 spectrometer using C_5_D_5_N with TMS as internal standard, and ESI-TOF mass on a Q-TOF-Micromass spectrometer, indicated that the compounds are ursolic acid (fraction A) and β-sitosterol (fraction B).

The fraction C was then added with NH_3_ (25%) to make it alkaline (pH 9) and then dissolved in chloroform with shaking. Finally, the chloroform phase was evaporated to obtain a total alkaloid extract (8 g), which was chromatographed on a silica gel column (3.5 ∞ 90 cm), using a linear gradient of CHCl_3_-MeOH system, and collected as 5 subfractions: 9.5-0.5, 9-1, 8.5-1.5, 8-2, and 7.5-2.5. These subfractions were filtered, concentrated and subjected to purification by TLC using precoated silica gel plates with CHCl_3_:MeOH:NH_3_ (50:50:3) solvent system. TLC separation of fractions demonstrated two bands with R_f_ of 0.33 and 0.63 of which the R_f_ 0.33 band showed antiviral activity and thus, identified by ^13^CNMR ^1^,HNMR and mass spectroscopy.

The article "An Indole Alkaloid from a Tribal Folklore Inhibits Immediate Early Event in HSV-2 Infected Cells with Therapeutic Efficacy in Vaginally Infected Mice" was retracted in 2025. Reasons: errors in the methods; duplicated images; duplicated data; duplicate publication.

### Cells and viruses

Vero cells (African green monkey kidney cells; ATCC, Manassas, VA, USA) were cultured in Dulbecco’s modified Eagle’s medium (DMEM) with 5-10% fetal bovine serum (FBS; Invitrogen, USA), 100 U/mL penicillin and 100 µg/mL streptomycin, at 37°C in 5% CO_2_. The viral strains used were HSV-2G (ATCC 734), purchased from the ATCC, along with the clinical isolates 1-4 and TK-deficient HSV-2, which were kindly provided by Professor P.K. Dutta and Professor M. Sengupta, Calcutta Medical College & Hospital, Kolkata, India. Virus stocks were prepared from infected culture at a multiplicity of infection (moi) of 0.5 for 1 h at 37°C. The residual viruses were then washed out with phosphate-buffered saline (PBS) and the cells were cultured for another 48-72 h. The cultured cells were lysed finally by three cycles of freezing and thawing, centrifuged at 1500 *g* at 4°C for 20 min and the collected supernatant was tittered by plaque assay, and stored at -80°C for further studies.

### Cytotoxicity assay

To determine the effect of fraction C and its isolated compound on uninfected cells, cultured Vero cells (10^4^ cells/well) in 96 well plates were exposed to various concentrations of the test drugs, in triplicate and incubated at 37°C in 5% CO_2_, using ACV and dimethylsulfoxide (DMSO, 0.1%) as controls. After 48 h, 10% 3-(4,5-dimethylthiazol-2-yl)-2,5-diphenyl tetrazolium bromide (MTT; Sigma) was added to each well with DMEM, incubated for 3-4 h, and then mixed with 100 µl of MTT solubilizing solution (Sigma), and the optical density (OD) was read by a plate reader at 570 nm with a reference wavelength of 690 nm. Data were calculated as the percentage of cell viability using the formula: [(sample absorbance-cell free sample blank)/mean media control absorbance)]X100%. The 50% cytotoxic concentration (CC_50_) causing visible morphological changes in 50% of Vero cells with respect to cell control was determined from the concentration-response curves after viable cell count [24].

### Antiviral and dose-response assay

In the antiviral assay Vero cell (10^4^ cells/well) culture on 96-well plates were infected with HSV-2G and the clinical isolates (0.5 moi) separately, and then exposed to the various concentrations of the test compound and ACV, in triplicate, and incubated for 72 h at 37°C in 5% CO_2_. The MTT assay was carried out, as described above and viral inhibition rate was calculated as: [(A_tv_-A_cv_)/(A_cd_-A_cv_)]X100%, where A_tv_ indicates the absorbance of test compound with virus-infected cells. A_cv_ indicates the absorbance of virus control, and A_cd_ the absorbance of the cell control. The antiviral concentration of 50% effectiveness (EC_50_) was defined as the concentration that achieved 50% inhibition of virus-induced cytopathic effects [24]. 

The article "An Indole Alkaloid from a Tribal Folklore Inhibits Immediate Early Event in HSV-2 Infected Cells with Therapeutic Efficacy in Vaginally Infected Mice" was retracted in 2025. Reasons: errors in the methods; duplicated images; duplicated data; duplicate publication.

For dose response assay the Vero cells were infected with HSV-2 isolates at 100-300 plaque-forming units (pfu) for 1 h at room temperature. Then the test compound at different concentrations (0-50 μg/ml) was added and the mixture was incubated at 37°C for 1-2 h, and virus yields were determined by plaque assay after 48 h of incubation [25]. The 50% inhibitory or effective concentration (EC_50_) was calculated from dose-response curves. Antiviral activities were also estimated by selectivity index (SI) calculated from CC_50_ and EC_50_ values.

### Plaque reduction assay

The Plaque reduction assay was used to evaluate the antiviral efficacy, using ACV and DMSO (0.1%) as positive and negative control respectively. Vero cell monolayers in twelve well plates, infected with wild type and clinical isolates of HSV-2 (100 pfu) were exposed to serial dilutions of test compound and then overlaid with 1% methylcellulose (Fluka, USA) to form plaques. The plaques developed after 72 h of incubation were fixed with 4% paraformaldehyde and stained with methylene blue (0.03%) in 70% methanol. The virus titers were calculated by scoring the plaque-forming units (pfu). The effective concentration of test compound that inhibited the number of viral plaques by 50-100% (EC_50_ and EC_100_) was interpolated from the dose-response curves [25]. 

### Time-of-addition assay

Following three different approaches, Vero cells in twelve well plate (4x10^5^) were exposed to the test compound (5.0 µg/ml) before infection, during infection or after infection with HSV-2G (100 pfu/well) at 0-24 h time intervals in triplicate, using DMSO (0.1%) and ACV (5.0 µg/ml) as controls. For pre-infection Vero cells were treated with the test compound either for 1 h or for 3 h, washed with PBS and then infected with HSV-2G in DMEM containing 2% FBS at 37°C. After 1 h adsorption the cells were covered with overlay media for plaque assay. For co-infection Vero cells were subsequently infected and treated with the test compound and after 1 h of incubation the virus-drug mixture was removed, washed with PBS three times, added with fresh media and subjected to the plaque assay. While for post-infection (p.i) the cells were infected with the virus first, allow to adsorb (1 h) and then treated with the test compound at intervals of 2, 3, 4, 5, 6, 8, 12, 24 h post infection. Finally the cells were harvested after 24 h for plaque assay [25].

The article "An Indole Alkaloid from a Tribal Folklore Inhibits Immediate Early Event in HSV-2 Infected Cells with Therapeutic Efficacy in Vaginally Infected Mice" was retracted in 2025. Reasons: errors in the methods; duplicated images; duplicated data; duplicate publication.

### Immunofluorescence assay

The HSV-2G (0.5 moi) infected Vero cell monolayer was treated with two different concentrations of the test compound (1.5 and 5.0 µg/ml) at 2 h and 4 h p.i, and washed twice with PBS to remove the cell debris. The cells were then fixed with paraformaldehyde (4%) and blocked with 1% bovine serum albumin (BSA) in 0.1% PBS-Triton X100 solution. The cells were further washed with PBS, then permeabilized with 0.1% Triton X100 in PBS, and incubated either overnight at 4°C or 1 h at room temperature with FITC-labelled polyclonal rabbit anti-HSV-2 antibody (Dako Cytomation, Denmark) to tag the drug treated virus. The cells were then washed with PBS and mixed with DAPI (Dako Cytomation, Denmark) to visualize both the virus and cell nucleus under Axio Imager M1 (Carl Zeiss, USA) inverted epifluorescence microscope [26]. 

### Attachment and penetration assay

To investigate whether the compound have any effect on viral adsorption or attachment, Vero cell monolayer in six well plate (10^6^) were prechilled at 4°C for 1 h and subsequently challenged with HSV-2G (200 pfu/well) in the presence of test compound (5.0 µg/ml), DMSO (0.1%) or ACV (5.0 µg/ml) for 3 h at 4°C. After infection, the wells were washed twice with ice-cold PBS to remove unbound virus, and overlaid with 1% methylcellulose to allow plaque formation. The plaques developed after 72 h of incubation were stained and counted [25,27]. 

For viral penetration assay prechilled (at 4°C for 1 h) Vero cell monolayer in six well plate were subsequently incubated with HSV-2G (300 pfu/well) for 3 h at 4°C to allow viral adsorption. The infected cells were then incubated with test compound (5.0 µg/ml), DMSO (0.1%) or ACV (5.0 µg/ml) for another 20 min at 37°C to facilitate viral penetration. At the end of the incubation period, extracellular non-penetrated virus was inactivated by citrate buffer (pH 3.0) for 1 min, and then the cells were washed with PBS and overlaid with overlay medium for plaque formation. The viral plaques developed after 48 h of incubation at 37°C were stained and counted [27].

### Virus inactivation assay

To determine the effect of test compound on the inactivation of virus particles, HSV-2G (10^4^ PFU/ml) was treated with the compound (5.0 µg/ml) at 37°C for 1 h and then, the mixture was 50 times diluted with fresh DMEM containing 2% FCS to yield sub-therapeutic concentration of the test compound. The virus inocula were then added to Vero cell monolayer. As a comparison, HSV-2G was mixed with the test compound, diluted immediately to 50-fold (no incubation period), and added to Vero cells for infection. The 50-fold dilution served to titrate the drugs below their effective doses and prevent meaningful interactions with the host cell surface. After adsorption for 1 h at 37°C, the diluted inocula were discarded, the cells were washed with PBS twice and then overlaid with overlay media and were subjected to the plaque assay, as described above [27,28].

The article "An Indole Alkaloid from a Tribal Folklore Inhibits Immediate Early Event in HSV-2 Infected Cells with Therapeutic Efficacy in Vaginally Infected Mice" was retracted in 2025. Reasons: errors in the methods; duplicated images; duplicated data; duplicate publication.

### Combined effect of test compound with Acyclovir

In order to analyze the combined effect of test compound (HM) and ACV on plaque formation the EC_50_ of both the agents as well as at various concentrations of the compounds against HSV-2G were tested and the combined effect was examined by plaque assay. Duplicate culture of Vero cells were infected with 100 PFU/0.2 ml of HSV-2G for 1 h and the cells were overlaid with 5 ml of overlay medium with various concentrations of HM and/or ACV and then incubated at 37°C for 72 h. The cells were then washed and fixed (4% paraformaldehyde) and stained with methylene blue (0.03%) to count the numbers of plaques for the determination of 50% inhibitory concentration of the plaque number from a curve, while the combined treatment was analyzed by isobologram method [29]. The EC_50_ was used to calculate the fractional inhibitory concentration (FIC) of the agents in combination. The interaction between test compound and ACV was interpreted according to the combined FIC index (FIC_compound_ + FIC_ACV_) as synergy (≤0.5), no interaction (0.5-4) or antagonism (>4).

### Western blot analysis

The HSV-2G (5 moi) infected Vero cells were treated with HM (5.0 µg/ml) at intervals of 2, 4, 6 and 8 h post-infection. After 24 h, equal amounts of protein (40 µg/sample) extract from whole cell were harvested in buﬀer (200 µl/well) containing 20 mM Tris (pH 7±0.5), 50 mM NaCl, 5% NP-40 and 0.05% DOC. The soluble fraction was then separated by centrifugation at 16000 g for 10 min at 4°C, subjected to SDS-PAGE and blotted to pre-equilibrated PVDF membrane (Thermo Scientific, USA). The membrane was then blocked in 5% NFDM in 1X TBST (20 mM Tris, pH 7.5, 150 mM NaCl, 0.5% Tween 20), rinsed and incubated with monoclonal anti-ICP4 or polyclonal anti-β actin (Shanta Cruz Biotech Inc., USA) antibody in 5% BSA at 4°C overnight. Immunoblotting was performed with peroxidase-labelled anti-rabbit polyclonal antibodies and visualized by ECL Western blot detection kit (Millipore, USA) [30]. 

### Quantitative real-time PCR

The HSV-2G (5 moi) infected Vero cells were treated with the test compound (1.5 and 5.0 µg/ml) for 2 h and 4 h intervals, and RNA was isolated immediately using RNeasy Mini kit (QIAGEN) following the manufacturer’s protocol. Then the total RNA (0.1 mg/ml) in RNase-free water in 20 µl of RT mix (containing 5X VILO Reaction Mix, 10X SuperScript Enzyme Mix and DEPC treated water) was subjected to cDNA synthesis using the GeneAmp PCR System 9600 (Perkin Elmer Corp, USA). The real-time PCR was performed with these products by using SYBR Green PCR Master Mix (Qiagen) following manufacturer protocol in a ABI Prism 7000 sequence detection system (Applied Biosystems, CA, USA). The PCRs were amplified at cycling conditions of: 95°C for 10 min and 40 cycles (15 s at 95°C, then 60 s at 60°C) in triplicate [31]. The sequences of primers used were as follows: ICP4 (5'-GACGTTGTGGACTGGGAAG-3' and 5'-ACTTAATCAGGTCGTTGCCG-3'); ICP27 (5'- CCTTTCTCCAGTGCTACCTG-3' and 5'-GCCAGAATGACAAACACGAAG-3') and GAPDH (5'-AAGGTCGGAGTCAACGGATT-3' and 5'-CTGGAAGATGGTGATGATGGGATT-3').

The article "An Indole Alkaloid from a Tribal Folklore Inhibits Immediate Early Event in HSV-2 Infected Cells with Therapeutic Efficacy in Vaginally Infected Mice" was retracted in 2025. Reasons: errors in the methods; duplicated images; duplicated data; duplicate publication.

### Electrophoretic mobility shift assay

Oligonucleotide sequence 5′-GCATGCTAATGATATTCTTTG-3′ of the ICP0 promoter of HSV-2G was biotinylated using Biotin 3' end DNA labelling Kit (Thermo Scientific, USA). The nuclear extracts of HSV-2G infected Vero cells treated with the test compound (5.0 µg/ml) or DMSO (0.1%) for 2 and 4 h intervals were prepared. Reaction mixtures (20 μl) contained, in addition to 3 μg of nuclear extracts, 20 fmol of Biotin 3' end-labelled probe, 50 ng/μl of poly (dI-dC), 2.5% glycerol, 0.05% NP-40 (1%), 5 mM MgCl_2_, and 1X binding buffer. After incubation for 20 min at room temperature, reaction mixtures were applied to 4% polyacrylamide gels in 0.5X Tris-borate-EDTA (TBE) buffer at 4°C. The gel was then transferred to Nylon membranes using Semi Dry Transfer Cell (Bio-Rad, USA), and transferred oligos were immobilized by UV cross-linking for 10 min. For detection of bound oligos, membranes were blocked with blocking buffer followed by addition of Streptavidin-Horseradish Peroxidase conjugate and developed according to the manufacturer’s instructions (Thermo Scientific, USA) [32]. For supershift assays nuclear extracts were pre-incubated with HCF-1 polyclonal antibodies for 30 min on ice.

### Co-immunoprecipitation assay

The HSV-2G infected, untreated or test compound treated (5.0 µg/ml) cells for 4 h were washed with ice-cold PBS and then lysed in a solution containing 10 mM Tris (pH 8.0), 170 mM NaCl, 0.5% NP40 and protease inhibitors for 30 min on ice with subsequent three freeze/thaw cycles at -80°C to lyse the nuclei. Cell debris was then removed by centrifugation and the supernatants were precleared with protein A-coupled Sepharose beads for 2 h. The lysates were then immunoprecipitated with HCF-1 or LSD1 antibodies as well as isotype-matched control antibodies plus protein A-Sepharose for at least 4 h or overnight. Beads were washed four times with 1 ml of wash buffer (200 mM Tris at pH 8.0, 100 mM NaCl and 0.5% NP-40), once with ice-cold PBS and boiled in 2X loading buffer. Finally the proteins were resolved by SDS-PAGE before probed with indicated antibodies [33].

The article "An Indole Alkaloid from a Tribal Folklore Inhibits Immediate Early Event in HSV-2 Infected Cells with Therapeutic Efficacy in Vaginally Infected Mice" was retracted in 2025. Reasons: errors in the methods; duplicated images; duplicated data; duplicate publication.

### *In vivo* Toxicity study

Male and female BALB/c mice (18-20 gm), acclimatized for 7-10 days with standard food and water *ad libitum*, housed in polypropylene cages in Animal House facility were used in accordance with the OECD guidelines accepted by the Committee for the purpose of control and supervision on experiments on animals (CPCSEA), Thiruvanmiyur, Chennai, India and as per the approval of the Institutional Animal Care and Use Committee (IACUC) of the Jadavpur University, Kolkata (Approval No: 367/01/C/CPCSEA). When required, the surgical procedures performed under Ketamine hydrochloride (100 mg/kg i.m.) anesthesia, and all efforts were made to minimize suffering. 

For acute toxicity studies, different concentrations of the test compound were administered orally to healthy 7-week-old BALB/c male or female mice, three times daily for 7 days, while for subacute toxicity study the animals were feed with the daily doses of the compound for 28 days. The control group (n=10) received normal saline, whereas the experimental groups (six groups, n=6) were administered with different doses of (25-150 mg/kg body weight) of the test compound and observed continuously for 72 h and then daily upto 30 days to record any change in weight, behaviour, sign of clinical toxicity or morbidity, and the LD_50_ of test compound was calculated by the method of Reed and Muench [34]. During the acute toxicity study, when required cervical dislocation was used to euthanize animals and the criteria for euthanasia were (i) severe illness or the animals in a moribund state (ii) severe pain and respiratory distress (iii) abnormal vocalisation, aggressiveness, posture and movements (iv) self-induced trauma (v) rapid weight loss, severe dehydration and significant bleeding. 

The mortality was calculated on the 30^th^ day, using weights and mortality data. Moreover, fresh blood was collected for the estimation of hematological and serum biochemical parameters by cardiac puncture, and then sacrificed to collect liver spleen and kidney for histopathological examination.

### Preparation and stability test of ointment formulation

The ointment of HM was prepared to evaluate its efficacy, in comparison with ACV ointment (5%, Cipla Ltd., Mumbai, India). The HM (25 and 50 mg) was mixed with simple ointment base, (100 g of petroleum jelly, Vaseline ^TM^), by gentle trituration to get homogenized ointment of 0.25% and 0.5% w/w of active compound. To obtain the most stable ointment, the stability was evaluated at accelerated conditions as per the guidelines of the International Conference on Harmonization on Stability testing of New Drug Substances and Products, 27^th^ October 1993. Further, the ointment samples were kept at different temperatures (40°C, 37°C, room temperature) for 45 days and observed periodically for physical changes like phase separation, development of objectionable color, odour, consistency etc. The accelerated deterioration of ointments was also evaluated by centrifugation at 10,000 rpm for 10 min [35]. The ointment samples resistant towards physical stability and centrifugation were also tested for spreadability by modified wooden block apparatus method [36]. The ointments were freshly prepared on every 5^th^ day.

The article "An Indole Alkaloid from a Tribal Folklore Inhibits Immediate Early Event in HSV-2 Infected Cells with Therapeutic Efficacy in Vaginally Infected Mice" was retracted in 2025. Reasons: errors in the methods; duplicated images; duplicated data; duplicate publication.

### Skin irritation test

To test the dermal hypersensitivity and related allergic manifestation of HM in ointment dosage form, three batches of female Balb/C mice (n=10) were used. About 20 mg of the HM ointment (0.5% w/w) or Vaseline base was applied on the shaved and cleaned dorsal area (100-150 mm^2^ area) of each animal. After 4 h the residual ointment was removed with warm water and blotted dry to observe the sign of inflammation and related redness, flash, flare and wheel correspond to hypersensitivity. For further confirmation of dermal toxicity of the test compound dorsal hair of Balb/C female mice (n=10) was shaved, removed with hair remover cream (Anne French, Wyeth Ltd., India), cleaned with luke warm water and dried with tissue paper. Then the naked skin (100-150 mm^2^ area) was abraded with a dermal (Seven-Star) needle and 0.1 g of ointment (0.25, 0.5%) was applied to the abraded area of cohorts of animals (n = 6). After 24 h the ointment was removed, washed with warm water and the animals were examined for erythema and edema within another 1 h. The animals were also observed upto the next 72 h for additional confirmation of toxicity.

### HSV-2 genital herpes in mice

Seven weeks old BALB/c female mice (n=6) were injected subcutaneously in the neck ruff with 100 µl of depo-medoxyprogesterone acetate (Sigma, USA) at 2 mg/mouse 5-7 days prior to infection to synchronize the estrus-cycle of the animals and facilitate infection. The HSV-2G stock was diluted and 10 µl of diluted suspension was inoculated to the vagina of each mouse by a sterile blunt ended micropipette tips. The mice were observed for 12 days to record the development of vaginitis or lethality. During this study, the intravenous (i.v.) administration of sodium pentobarbital (18% of 200 mg/kg) in a dose of 200 mg/kg was used to euthanize the animals showing the signs of severe illness or a moribund state, considering the following factors: (i) signs of severe pain and respiratory distress (ii) abnormal vocalisation, aggressiveness, posture and movements (iii) self-induced trauma (iv) rapid weight loss, severe dehydration and significant bleeding (v) skin ulceration with pain (vi) severe swelling including redness of vagina and its surrounding tissues along with hair loss in the genital area (vii) hind limb paralysis or other factors related to the animals in severe pain or distress. The median lethal dose (LD_50_) was determined to be equal to 9 X 10^4^ pfu [37].

The article "An Indole Alkaloid from a Tribal Folklore Inhibits Immediate Early Event in HSV-2 Infected Cells with Therapeutic Efficacy in Vaginally Infected Mice" was retracted in 2025. Reasons: errors in the methods; duplicated images; duplicated data; duplicate publication.

### Therapeutic Efficacy of Oral and Topical Application of HM in Mice

Seven week old acclimatized female BALB/c mice were divided into two separate batches, each with five groups (n=20). First group served as control, while the groups II-V of both the batches were injected subcutaneously in the neck ruff with 100 µl of depo-medoxyprogesterone acetate (Sigma, USA) at 2 mg/mouse, 5-7 days prior to infection to synchronize the estrus-cycle and facilitate infection. The vaginal area of each animal was swabbed with calcium alginate and then inoculated with HSV-2G at 9 X 10^5^ pfu (10 LD_50_) in 10 µl volume, intravaginally with a blunt ended micropipette tips. After 3-4 h of viral inoculation the animals of group III and IV were treated orally with HM (0.25 and 0.5 mg/kg) and the group V with ACV (5 mg/kg body weight), twice for 7 successive days; while group II was served as infection control. Finally, five animals from each group (I-V) of the first batch were sacrificed on day 2, 4, 6 (during the treatment schedule), and 8^th^ day (one day after complete treatment) for the determination of viral load. The collected samples were homogenized in PBS, centrifuged at 3000 rpm for 15 min and the virus yield in the supernatant was determined by plaque assay. The infected vaginal tissues from untreated and treated animals were collected for histopathological study as described above [37]. On the otherhand, the second batch of five groups (n=20) including control, infected, as well as infected and drug treated animals were observed for another twelve days, after the completion of treatment schedule, for the development of vaginitis or lethality. Genital pathology following HSV‐2 challenge was monitored daily and scored on a five-point scale: no signs of infection (0); slight redness of external vagina (1); swelling and redness of external vagina (2); severe swelling and redness of both vagina and surrounding tissue along with hair loss in the genital area (3); hind-limb paralysis (4); and death (5).

To test the efficacy of HM or ACV ointments the animals were infected with HSV-2G (9 X 10^5^ PFU), as described above. Following inoculation, a vaginal sample were collected from each animal by sterile cotton swab and transferred to 0.5 ml of PBS and stored at -20°C. The mice were divided into six groups (n=20) including two test groups (0.25 and 0.5% HM ointment) and one each of ACV control (5% ointment), vehicle control (ointment base), no treatment (virus control) and uninfected control group. Symptoms of viral vaginitis including topical edema of the vaginal tract with turbid secretions were observed on the third day of infection. Treatment starts on day 3 post-infection by applying 2 mg of ointment per mouse, twice daily for 7-days to the vaginal tract with sterile cotton swabs. The infected mice were observed for at least 30 days to determine their mortality and the number of days for mortality. The vaginal swab samples were obtained one day following the completion of the treatment, and from the deceased animals immediately following their death. The samples were then diluted five times in MEM and used to infect Vero cells. Samples that gave positive cytopathic effects were considered positive for HSV-2 [37]. Moreover, to assess the viral shedding, vaginal washes from infected mice were collected, diluted with fresh media, and then infected to Vero cells in six-well plates to determine the virus yield by the plaque reduction assay [37]. During the therapeutic efficacy study of the test compounds, sodium pentobarbital was administered i.v. to euthanize the animals showing the same signs and factors considered during the viral LD_50_ determination. 

The article "An Indole Alkaloid from a Tribal Folklore Inhibits Immediate Early Event in HSV-2 Infected Cells with Therapeutic Efficacy in Vaginally Infected Mice" was retracted in 2025. Reasons: errors in the methods; duplicated images; duplicated data; duplicate publication.

### Statistical analysis

The antiviral activity of test compound was expressed as a therapeutic or selectivity index (SI), determined as the ratio of CC_50_ to EC_50_. In general, an SI greater than 4 is indicative of positive anti-viral activity, while compounds having SI values of 10 or more was evaluated for anti-viral activity spectrum. The statistically different effects of test compound or ACV on viral inhibition were compared with the control group or among test drugs using the Student’s t-test. While the dose-dependent effect of the test compound was determined by linear regression. Statistical analysis of toxicity and efficacy studies of test compound on different batches were done by one way ANOVA or Student’s t-test.

## Results

### Isolation and identification of an antiviral compound from *O. nicobarica*

The alcoholic extract was filtered and solvent-evaporated to a powdered residue (32 g). The residue was suspended in water and extracted with n-butanol by repeated Silica-gel CC, and subsequently eluted with PE, PE:CHCl_3_, CHCl_3_, CHCl_3_:MeOH and MeOH, which yielded three fractions A, B and C. Fractions A and B were isolated and identified as ursolic acid and β-sitosterol by spectroscopic analysis [24]. The bioactive fraction C (8 g) was further chromatographed on silica gel column (3.5 ∞ 90 cm), with CHCl_3_:MeOH solvent system, concentrated, purified and isolated into two sub-fractions by TLC using CHCl_3_:MeOH:NH_3_ (50:50:3) solvent system. The sub-fraction with Rf 0.33 was found to inhibit HSV-2 in cell cultures and thus, purified by repeated CC and characterized by physical and spectroscopic analyses. The ^1^H and ^13^C NMR spectra (Figure S1A-D), and ESI-TOF mass (Figure S1E) revealed that the compound (compound-XX) having ESI-TOF MS (positive): *m*/*z* 215[M+H]^+^; ^1^H NMR (C_5_D_5_N):δ 11.4(s), 7.54(d, *J*=8.4Hz), 7.29(d, *J*=2.4Hz), 6.99(dd, *J*=8.4,1.8 Hz), 3.86(dt, *J*=9.0,1.2 Hz), 3.71(s), 2.93(t, *J*=9.0Hz); and ^13^C NMR: δ 165.5(s), 161.9(s), 144.2(s), 126.9(s), 124.8(d), 123.2(d), 119.9(s), 115.1(d), 94.9(d), 55.8(q), 42.6(t), 19.8(t), 19.4(q) is 7-methoxy-1-methyl-4,9-dihydro-3*H*-pyrido[3,4-*b*]indole (HM, Figure S1F). Physicochemically HM was a light yellow powder, with melting point 229°C and boiling point 120-140°C, slightly soluble in basic water but soluble in DMSO, having the chemical formula of C_13_H_14_N_2_O, Molecular Mass 214.3 g/mol and pKa 9.8 (Figure S1F). 

The article "An Indole Alkaloid from a Tribal Folklore Inhibits Immediate Early Event in HSV-2 Infected Cells with Therapeutic Efficacy in Vaginally Infected Mice" was retracted in 2025. Reasons: errors in the methods; duplicated images; duplicated data; duplicate publication.

### Assessment of cytotoxicity and anti-HSV efficacy of the isolated HM

Cellular viability assays, presented in Table 1, revealed that HM exhibited cytotoxicity (CC_50_) against Vero cells at 30 µg/ml, which is much higher than their EC_50_ (1.1-1.7 μg/ml) against HSV-2G and other isolates, indicating significant antiviral activity, compared to ACV (2.9-5.2 µg/ml). Interestingly the TK deficient strain had EC_50_ of >30 against ACV but sensitive to HM at only 2.8 µg/ml. Furthermore, the SI index of HM against the tested strains indicated its activity against HSV-2. 

**Table 1:** Assessment of cytotoxicity and anti-HSV-2 activity of HM.

Virus	HM (µg/ml)			Acyclovir (µg/ml)		
	CC_50_^a^	EC_50_^b^	SI^c^	CC_50_^a^	EC_50_^b^	SI^c^
HSV-2G (ATCC 734)	30	1.5 ± 0.1	20.0	130	2.9 ± 0.1	44.8
Clinical Isolate 1		1.7	17.6		3.5	37.1
Clinical Isolate 2		1.5	20.0		3.1	41.9
Clinical Isolate 3		1.1	27.3		5.2	25.0
Clinical Isolate 4		1.6	18.7		4.4	29.5
TK deficient strain		2.8	10.7		>30	-

a The 50% cytotoxic concentration (CC_50_) for Vero cells.

b Concentration(s) of HM producing 50% inhibition (EC_50_) of virus-induced cytopathic effect of three separate experiments.

c Selectivity index (SI) = CC_50_/EC_50_

In order to understand the quantitative and temporal aspects of the antiviral activity of HM, we conducted plaque reduction assays. The results showed that HM inhibited both the wild type and clinical isolates of HSV-2 in a dose-dependent manner, and maximum (>99%) inhibition of plaque formation was observed at 5.0 µg/ml (Figure 1A). On the otherhand, ACV showed 77.9% inhibition of plaque formation against HSV-2 at 5.0 μg/ml, but no inhibition was noticed with 0.1% DMSO, used as solvent (data not shown). Interestingly, HM also showed 60-80% plaque inhibition of the clinical isolates tested.

The article "An Indole Alkaloid from a Tribal Folklore Inhibits Immediate Early Event in HSV-2 Infected Cells with Therapeutic Efficacy in Vaginally Infected Mice" was retracted in 2025. Reasons: errors in the methods; duplicated images; duplicated data; duplicate publication.

**Figure 1:** Anti-HSV efficacy of HM. [A] **Plaque** **Reduction** **Assay**. Infected cells were treated with HM or ACV at 0.5-50 μg/ml, overlaid with methylcellulose and plaques developed after 2-3 days were stained. The % of plaque number reduction was calculated, and the effective concentration of drug that inhibited the number of viral plaques was interpolated from the dose-response curve. [B] **Time** **course** **analysis**. Inhibitory effects of HM and ACV at various time points prior to infection (-3 to -1 h), at the time of infection (0 h) and post-infection (2-24 h) with HSV-2 were evaluated by plaque reduction assay. Each bar represents the mean ± S.E.M of three independent experiments.

To investigate the activity of HM on viral infection cycle we performed the time-of-addition assay. Addition of HM (5.0 µg/ml) to HSV-2G infected Vero cells at different time points revealed that HM was effective at 2-4 h post-infection, whereas no inhibition was found when virus particles were exposed to HM before infection (pre-infection) or at the time of infection (co-infection). These findings suggested that the antiviral activity of HM was not due to the inhibition of viral adsorption or entry to the host cell but the interference with the immediate early replication of HSV-2 (Figure 1B). 

Further, to confirm the antiviral activity of HM we performed an independent IFA of virus-infected Vero cells treated with HM (1.5 and 5.0 µg/ml) for different time points and tagged with specific anti-HSV-2 antibodies. The results demonstrated that HM was most effective in reducing the number of infected fluorescent cells when added to the cultures at 4 h post-infection (Figure 2), but not in infected untreated control.

**Figure 2:** Immunofluorescence studies of HSV-2 infected cells treated with HM. Cells treated with HM at 2-4 h post-infection (p.i) were fixed with paraformaldehyde and blocked with BSA-PBS-triton X100 solution. After permeabilization, cells were incubated with FITC-labelled polyclonal rabbit anti-HSV-2 antibody, and observed under Axio Imager M1 (Carl Zeiss, NY, USA) inverted epifluorescence microscope. Cell Control [a]; Cells treated with HM (5.0 μg/ml) at 2 h [b] and 4 h [c] p.i.; Virus control at 2 h p.i [d]; infected cells treated with HM at 1.5 μg/ml [e], and 5.0 μg/ml [f] at 2 h p.i; Virus Control at 4 h p.i [g]; infected cells treated with HM at 1.5 μg/ml [h] and 5.0 μg/ml [i] at 4 h p.i.

The article "An Indole Alkaloid from a Tribal Folklore Inhibits Immediate Early Event in HSV-2 Infected Cells with Therapeutic Efficacy in Vaginally Infected Mice" was retracted in 2025. Reasons: errors in the methods; duplicated images; duplicated data; duplicate publication.

As the time of addition assay and IFA indicated that HM inhibited HSV-2 at 2-4 h post-infection, i.e., the early event of viral life cycle, including attachment and penetration, we investigated these steps separately. Result presented in Figure 3A showed that HM had no effect on HSV-2 attachment or penetration into Vero cells (Figure 3B), like ACV, indicating that HM was not inhibiting viral entry to the host cell. We then examined whether the efficacy of HM could increased in combination with ACV by the drug combination assay. The antiviral activity of various combinations of HM and ACV, using the isobologram method, failed to demonstrate any additive or synergistic interaction of combined therapy, with the FIC index of 0.92 (Table 2). 

**Figure 3:** Effect of HM and ACV on HSV-2 attachment and penetration. [A] **Attachment** **assay**: Prechilled cells at 4°C for 1 h were infected with HSV-2G (200 pfu) and then untreated or treated with HM. After incubating at 4°C for another 3 h, the medium was aspirated, washed and overlaid with methylcellulose to form plaques. The plaques developed after 72 h were stained and counted. [B] **Penetration** **assay**: Prechilled cells at 4°C for 1 h was infected with HSV-2G (300 pfu) for 3 h at 4°C and then untreated or treated with HM (5µg/ml) or DMSO (0.1%), and incubated for 20 min at 37°C to facilitate viral penetration. Then the extracellular non-penetrated virus was inactivated by citrate buffer (pH 3.0) for 1 min, washed with PBS and overlaid with overlay medium to form plaques. The plaques developed were then stained and counted.

**Table 2:** Inhibitory effects of HM in combination with Acyclovir.

Compound	EC_50_	FIC_compound_ + FIC_ACV_	Inhibitory effect
	HSV-2	HSV-2	
Isolated HM alone	1.5 ± 0.1	-	-
Acyclovir alone	2.9 ± 0.1	-	-
Acyclovir + HM	0.73 ± 0.1	0.92	No interaction

The interaction between HM and ACV was interpreted according to the combined FIC index [FIC_compound_ + FIC_ACV_] as synergy (≤0.5), no interaction (0.5 - 4) or antagonism (>4) (32).

### Effect of HM on HSV-2 immediate early gene expression

Then to determine how the test compound interfere with the early steps of HSV-2 infection in Vero cells, we investigated the immediate early (IE) gene expression of the virus in presence of HM. Briefly, the HSV-2 infected Vero cells were treated with HM (5.0 µg/ml) at different time point (2-8 h) and the whole cell extract was used for the detection of ICP4 level by Western blot analysis (Figure 4A), as ICP4 is an essential factor for early and late promoters. Interestingly, we observed a significant decrease of ICP4 levels in HM treated cells upto 6 h post-infection. On the otherhand, the quantitative real-time PCR analysis indicated a significant decrease of the copy number of IE proteins ICP4 and ICP27 (essential for efficient expression of late gene products) at 1.5 and 5.0 µg/ml, in time dependent manner (Figure 4B). 

The article "An Indole Alkaloid from a Tribal Folklore Inhibits Immediate Early Event in HSV-2 Infected Cells with Therapeutic Efficacy in Vaginally Infected Mice" was retracted in 2025. Reasons: errors in the methods; duplicated images; duplicated data; duplicate publication.

**Figure 4:** Effect of HM on IE gene expression. [A] **Western** **blot** **analysis**: 40 µg of protein sample from whole cell extracts were separated by SDS-PAGE, blotted to nitrocellulose, and filters were incubated with monoclonal anti-ICP4 or polyclonal anti-β actin antibody followed by decoration with peroxidase-labelled anti-rabbit polyclonal antibodies, respectively and visualized using ECL Western blot detection kit. [B] **Quantitative** **real** **time** **PCR**: HSV-2G (5 moi) infected cells were treated with HM (5.0 µg/ml) for 2 and 4 h. After incubation at 37°C RNA was isolated and subjected to cDNA synthesis. Then quantitative real-time PCR was performed with these products by using SYBR Green PCR Master Mix. PCRs were amplified with the cycling conditions of: 95°C for 10 min and 40 cycles (15 s at 95°C, then 60 s at 60°C).

### HM down regulates transcription of HSV-1

Next, we investigated the effect of HM on the IE transcriptional events, by EMSA and supershift assay of the binding of IE complex on ICP0 promoter of HSV-2. The results, presented in Figure 5A, showed that the binding of IE complex on ICP0 promoter was reduced in drug treated cells at 4 h post-infection, indicating that HM interfered in the recruitment of Vp16-HCF-1-Oct-1 complex on TAATGARAT region of ICP0 promoter, leading to the decreased viral transcription. Further, the supershift assay indicated that HM affected the interaction of HCF-1, a component of IE complex (Figure 5B). 

**Figure 5:** Effect of HM on viral IE transcriptional events. [A] **EMSA**: HSV-2G infected Vero cells were treated with HM for 2 and 4 h and assayed for EMSA. Biotin-labelled oligo was present in Lanes 1-6; P, biotin labelled oligo, M, mock control. [B] **Supershift** **assay**: nuclear extracts from HSV-2G infected HM treated cells for 4 h p.i. was pre-incubated with HCF-1 polyclonal antibodies, added with reaction mixture, applied to non-denaturing 4% polyacrylamide gels and visualized by autoradiography. P, free biotin labelled probe; ns, nonspecific binding. [C] HCF-1 or LSD1 were immunoprecipitated in HM treated virus infected Vero cell lysate and the association was confirmed by immunoblotting with anti-HCF-1 and anti-LSD1 antibodies.

The article "An Indole Alkaloid from a Tribal Folklore Inhibits Immediate Early Event in HSV-2 Infected Cells with Therapeutic Efficacy in Vaginally Infected Mice" was retracted in 2025. Reasons: errors in the methods; duplicated images; duplicated data; duplicate publication.

Recently, it has been demonstrated that HCF-1-dependent recruitment of LSD1 plays an important role in the initiation of HSV-2 infection [33]. Therefore, we further investigated the effect of HM on the association of HCF-1 with LSD1 in infected cells, by co-immunoprecipitation study. The whole cell lysates of the infected cells (4 h. p.i.), treated or untreated, were immunoprecipitated with an anti-HCF-1 or LSD1 polyclonal antibody followed by immunoblotting with LSD1 or HCF-1 antibody. Interestingly, we observed that the infected cells treated with HM (5.0 µg/ml) have weak or no co-immunoprecipitation at 4 h p.i., indicating a poor association between HCF-1 and LSD1; whereas the association was strong in the infected untreated cells (Figure 5). Thus, the significant reduction of interaction between HCF-1 and LSD1 in HM treated cells confirm that HM interfere with the LSD1 recruitment.

### *In vivo* Toxicity Studies

Acute toxicity studies revealed that HM was safe up to 50 mg/kg body weight without any obvious toxicity in mice, and the LD_50_ was 132.5 mg/kg. Moreover, subacute toxicity studies showed no significant change in haematological and biochemical parameters including SGOT and SGPT level or any histopathological changes in major organs of the treated mice upto 30 days (data not shown). Furthermore, the skin irritation test showed that HM was safe at both 0.25 and 0.5% doses.

### HSV-2 Genital herpes in Mice

The therapeutic efficacy of HM, presented in Figure 6, was examined in mice infected with HSV-2G intravaginally and monitored the development of lesions by scoring on a five point scale. The virus yields in the vaginal tissue and brain from infected mice on day 2, 4 and 6 after infection, showed that HM reduced HSV-2 yield in a dose and time response manner. In the vaginal mucosa the virus yield was 85.18, 84.70, and 78.8% with HM 0.25 mg/kg, while it was 77.8, 76.4 and 54.9% at 0.5 mg/kg on day 2, 4 and 6, respectively. On the otherhand, the reduction in brain was 73% and 65.4% on day 4, while it was 58.7% and 50.4% on day 6. Interestingly, for acyclovir the yield was 45.4% in vaginal mucosa and 59.1% in brain. Thus, our results exhibited potent anti-HSV-2 activity of HM by reducing lesion score and virus yield in vaginal mucosa as well as in brain (p<0.01) of the infected animals.

**Figure 6:** *In* *vivo* efficacy of HM. BALB/c mice were fed with HM (0.25 or 0.5 mg/kg) or ACV (5 mg/kg) and after 8 h of drug treatment the animals were infected with HSV-2G (9 X 10^5^ pfu per animal) intravaginally. The challenged animals of test groups were fed with HM twice daily for 7 days. Development of lesions and death were observed three times daily, while brain and vaginal tissue were collected after sacrification on days 2, 4, 6 or 8 after infection, homogenized and centrifuged. The supernatant was used for the determination of virus yield by plaque assay. Mean lesion score [A], Mean±S.D. of virus yield at log_10_ (PFU/organ) in vaginal tissue [B] and brain [C].

The article "An Indole Alkaloid from a Tribal Folklore Inhibits Immediate Early Event in HSV-2 Infected Cells with Therapeutic Efficacy in Vaginally Infected Mice" was retracted in 2025. Reasons: errors in the methods; duplicated images; duplicated data; duplicate publication.

Further, the histopathology of vaginal tissues of animals revealed that the uninfected vaginal tissue had intact vaginal epithelium without any inflammation and infection (Figure 7A). While the HSV-2G infected genital tissues showed acute inflammation and leukocytic infiltration with extensive infection (Figure 7B). Interestingly, the infected animals treated with HM (0.5 mg/kg) and ACV (5 mg/kg) demonstrated limited infection (Figure 7C, D). 

**Figure 7:** Histopathology of Genital tissue of Balb/C mice : uninfected [A], infected with HSV-2G [B], HSV-2G infected animals treated with 0.5 µg/ml of HM [C], and ACV at 5 µg/ml [D].

### Therapeutic effects of HM ointment(s) in genital HSV-2 infected mice

Three days following HSV-2G inoculation, all animals except the uninfected control group developed symptoms of vaginitis. The infected untreated animals (virus control) showed a very low survival rate and time (Table 3), similar to the animals of ointment base control. In contrast, the survival rate for the HM (0.5%) and ACV (5%) treated group was 70 and 80% respectively. The six dead animals in HM treated group lived for an average of 11.15 days, signiﬁcantly longer than those in the virus control group, indicating that the animals that received 0.5% HM ointment had nearly similar survival rate and time to the ACV treated group. The HSV-2 was detected in the vaginal samples from all animals, except the uninfected control group, following inoculation, conﬁrming that the animals were infected (Table 3). Further, the samples recovered from the animals following treatment or post-mortem was positive for HSV-2. Interestingly, the number of samples positive for HSV-2 was similar to the number of death, except in the HM ointment groups, where the number of HSV-2-positive samples was considerably higher than the number of death. Moreover, the plaque assay of vaginal washes, collected to determine virus shedding, showed no virus in ACV or HM treated animals from day 7, indicating the efficacy of the test compound.

**Table 3:** Efficacy of HM ointment in HSV-2 genital infection model.

Drug Treatment	No. of animals	No. of animals survived	No. of death	Survival (%)	Days-to-mortality (mean±S.D. days)^a^	No. of vaginal samples containing HSV-2	
						Before treatment	After treatment/death
HM 0.5%	20	14	06	70*^b^	11.15 ± 2.34*	20	07*
HM 0.25%	20	09	11	45*	9.45 ± 2.66*	20	15*
ACV 5%	20	16	04	80*	11.85 ± 1.33*	20	05*
Vaseline Base	20	02	18	10**	7.65 ± 2.87**	20	18**
Virus control	20	01	19	5	6.75 ± 1.93	20	19
Uninfected	20	20	0	100	NA^c^	0	0

a Average time for mortality to occur following infection.

^b^ P value from t-test between test group and virus control group. * P > 0.01; ** P < 0.05

c Not applicable.

The article "An Indole Alkaloid from a Tribal Folklore Inhibits Immediate Early Event in HSV-2 Infected Cells with Therapeutic Efficacy in Vaginally Infected Mice" was retracted in 2025. Reasons: errors in the methods; duplicated images; duplicated data; duplicate publication.

## Discussion

The present study demonstrated the *in vitro* and *in vivo* anti-HSV-2 activity of an alkaloid HM isolated from an ethnomedicinal herb *O. nicobarica*, used by Shompen and Nicobarese tribes of Nicobar group of Islands, India for skin ailments, along with its mode of action. In our previous studies, we reported the moderate anti-inflammatory [22] and antimicrobial [23] activities of this plant extract. However, the present phytochemical investigations of active extract revealed three fractions, of which fractions A yielded an antivirally weak triterpene ursolic acid, while the fraction B contain antivirally inactive β-sitosterol. Interestingly the purification of the most active fraction C yielded a pure alkaloid, identified as 7-methoxy-1-methyl-4,9-dihydro-3*H*-pyrido[3,4-*b*]indole (HM) by melting point ^1^,HNMR ^13^CNMR, and Mass spectral analysis. On the otherhand, the ursolic acid obtained from fraction A was less active compared to the fraction C and thus, we have not included ursolic acid for further study. 

The MTT and plaque reduction assay revealed that HM has strong antiviral activity against wild type as well as the clinical isolates of HSV-2 *in vitro* at non cytotoxic concentration with respect to its EC_50_ and selectivity index, compared to ACV. The plaque reduction assay demonstrated that HM inhibited HSV-2 infection in a dose-dependent manner, and > 99% inhibition was found at 5.0 µg/ml. In order to understand the quantitative and temporal aspects of the antiviral activity of HM we conducted kinetic studies. Addition of HM to virus infected cells at different time points revealed that HM was effective at 2-4 h post-infection. We further performed the immunofluorescence assay to determine the HM action on HSV-2 antigen expression, and observed that the maximum reduction of infected fluorescent cells occur at 4 h post-infection. This suggests that HM reduced > 99% of viral load at 4 h post infection, indicating its interference at an early stage of HSV multiplication. Further study showed that HM was unable to prevent the attachment or penetration of HSV-2, like ACV, suggesting that the mode of action of HM is not the prevention of viral adsorption or penetration, but perhaps the interference of early events of HSV replication, including the immediate early (IE) transcriptional events. Moreover, the drug combination study (HM ± ACV) did not reveal any additive or synergistic effects, suggesting that HM may work through similar targets but at different time points. 

The article "An Indole Alkaloid from a Tribal Folklore Inhibits Immediate Early Event in HSV-2 Infected Cells with Therapeutic Efficacy in Vaginally Infected Mice" was retracted in 2025. Reasons: errors in the methods; duplicated images; duplicated data; duplicate publication.

Next, to investigate the possible mode and mechanism of action of HM on early events of viral infection cycle we studied the effect of HM on IE gene expression of HSV-2. To study whether HM interferes any of the events of IE gene expression we measure the two major end products, ICP4 and ICP27 of IE gene by Western Blot and quantitative real-time PCR analysis. The results showed the reduced expression of both ICP4 and ICP27 in HSV-2 infected HM treated cells but not in untreated cells. It is known that during IE transcription the VP16 of HSV virion recruited several cellular coactivators including HCF-1 and Oct-1 on IE promoter to form the IE transcriptional complex for transactivation and synthesis of IE gene at 2-4 h post-infection [40]. Thus, we have studied the interaction of HM, if any, with the formation of IE transcriptional complex consisting of VP16, HCF-1 and Oct-1 by EMSA. The results revealed that HM indeed interact with the DNA-protein assembly leading to the reduced level of IE complex, and the treatment of HM in first 4 h after infection was more effective in preventing the binding of HCF-1-VP16-Oct-1 complex on ICP0 promoter. Further, the supershift assay showed that the expression of HCF-1 was reduced in presence of HM. Next, we investigated the effect of HM on the association of HCF-1 with LSD1, a chromatin associated cofactor of host cell, in HSV-infected cells by co-immunoprecipitation study. It was known that HSV used HCF-1 to recruit LSD1 to its IE promoters during IE transcription [33]. Our data demonstrated that HM treated HSV-2 infected cells had weak or no precipitation reaction at 4 h p.i., indicating a poor association between HCF-1 and LSD1, whereas it was strong in the infected untreated cells. This observation is consistent with the report that HCF-1-dependent recruitment of LSD1 plays an important role in the initiation of HSV infection, and depletion or inhibiton of LSD1 activity by MAO inhibitors Pargyline and Tranylcypromine resulted in a block to viral IE gene expression with dose dependent decrease in viral IE proteins in HSV infected cells [33]. Thus, the significant reduction of interaction between HCF-1 and LSD1 in HM treated HSV-2 infected cells confirm that HM interfered with the recruitment of LSD1, a vital component of viral IE transcription. 

To know the safety profile of the test compound, we conducted animal toxicity study in Balb/C mice, and found that HM is moderately safe up to 50 mg/kg body weight with almost normal biochemical and haematological parameters, and without any detectable toxicity in major organs, compared to untreated control. The skin irritation test also revealed that HM at 0.25 and 0.5% dose is completely safe. Then we determined the *in vivo* efficacy of HM (oral and tropical) treatment in mice vaginally infected with HSV-2G. The results showed that the oral treatment of HM significantly reduced virus yields in the vaginal tissue and brain on day 4 and 6 after infection, compared to ACV and virus control(s), in a dose dependent manner, indicating that HM has strong anti-HSV-2 activity (p < 0.01). The results also revealed that the variation of virus yield percent on day 2-6 post infection was probably due to the differences in the distribution of HM in animal body after absorption or its affinity towards the central nervous system. Further, the therapeutic efficacy of topical application of HM is clearly evident in genital herpes model, as the HM ointment reduced both viral lesion and yield in a dose-dependent manner compared to the ointment base with no efficacy. Interestingly the therapeutic effect of HM (0.5%) ointment was nearly equivalent to 5% acyclovir ointment. Thus, this study for the first time, demonstrated that HM isolated from a folk medicine might have beneficial effects in preventing latency associated complications in the central nervous system due to HSV infection. 

The article "An Indole Alkaloid from a Tribal Folklore Inhibits Immediate Early Event in HSV-2 Infected Cells with Therapeutic Efficacy in Vaginally Infected Mice" was retracted in 2025. Reasons: errors in the methods; duplicated images; duplicated data; duplicate publication.

The available literature suggests that the isolated compound is similar to harmaline [38,39]. The harmaline is a well known CNS stimulant that inhibit acetylcholinesterase [40], histamine N-methyltransferase, and monoamine oxidase A [41] with vasorelaxant [38] and weak neurotoxic effect [40] in rats at higher dose [42]. However, our study demonstrated that HM has potential anti-HSV-2 activity in mice at 0.25 and 0.5 mg/kg b.w. (20 µg/animal), and even at a single dose of 50 mg/kg HM do not produce visible toxic effect on tested animals, probably because HM is less psychoactive than its related compounds [42].

In summary, we have isolated an alkaloid HM from a tribal folklore *O. nicobarica* having potent antiviral activity by interfering with the IE transcriptional event of HSV-2. Moreover, HM is well tolerated in mice at its antiviral dose and significantly reduced virus yield in mouse. As IE complex is a critical component of the reactivation mechanism of herpes viruses, our observations indicated that HM may prevent the multiplication and reactivation of the virus, and provide an interesting molecular target for the development of better drug to treat HSV-2 infections.

## Supporting Information

Figure S1 **NMR, mass spectra and structures of the isolated compound from *O. nicobarica*.**
(TIF)

The article "An Indole Alkaloid from a Tribal Folklore Inhibits Immediate Early Event in HSV-2 Infected Cells with Therapeutic Efficacy in Vaginally Infected Mice" was retracted in 2025. Reasons: errors in the methods; duplicated images; duplicated data; duplicate publication.

## References

[1] AkhtarJ, ShuklaD (2009) Viral entry mechanisms: cellular and viral mediators of herpes simplex virus entry. FEBS J 276: 7228-7236. doi:10.1111/j.1742-4658.2009.07402.x. PubMed: 19878306.19878306PMC2801626

[2] Sandri-GoldinRM (2006) Alpha Herpesviruses: Molecular and Cellular Biology. Caister Academic Press ISBN 978-1-904455-09-7.

[3] OstroveJM, LeonardJ, WeckKE, RabsonAB, GendelmanHE (1987) Activation of the human immunodeficiency virus by herpes simplex virus type 1. J Virol 61: 3726-3732. PubMed: 2446005.244600510.1128/jvi.61.12.3726-3732.1987PMC255985

[4] FelserJM, KinchingtonPR, InchauspeG, StrausSE, OstroveJM (1988) Cell line containing varicella-zoster virus open reading frame 62 and expressing the 'IE' 175 protein complement ICP4 mutants of herpes simplex virus type 1. J Virol 62: 2076-2082. PubMed: 2835512.283551210.1128/jvi.62.6.2076-2082.1988PMC253298

[5] GiusD, LaiminsLA (1989) Activation of human papillomavirus type 18 gene expression by herpes simplex virus type 1 viral transactivators and phorbol ester. J Virol 63: 555-563. PubMed: 2536091.253609110.1128/jvi.63.2.555-563.1989PMC247723

[6] CoreyL, WaldA, CelumCL, QuinnTC (2004) The effects of herpes simplex virus-2 on HIV-1 acquisition and transmission: a review of two overlapping epidemics. J Acquir Immune Defic Syndr 35: 435-445. doi:10.1097/00126334-200404150-00001. PubMed: 15021308.15021308

[7] KhandelwalM (2006) Genital herpes complicating pregnancy. Obstet Gynecol 107(3): 740‐7411. doi:10.1097/01.AOG.0000202543.49213.6c. PubMed: 16507951.16507951

[8] HabifT (2004) Warts, Herpes Simplex, and Other Viral Infections. Clinical Dermatology, 4th Edition HabifT New York: Mosby pp. 381-388.

[9] MayaudP, McCormickD (2001) Interventions against sexually transmitted infections (STI) to prevent HIV infection. Br Med Bull 58: 129-153. doi:10.1093/bmb/58.1.129. PubMed: 11714628.11714628

[10] ShuyunS, KelongH, YupingZ, YuZ, QizhenD (2007) Purification and identification of antiviral components from *Laggera* *pterodonta* by high-speed counter-current chromatography. J Chromatogr 859(1): 119-124.10.1016/j.jchromb.2007.09.01617920342

[11] NagotN, OuédraogoA, FoulongneV, KonatéI, WeissHA et al. (2007) Reduction of HIV-1 RNA levels with therapy to suppress herpes simplex virus. N Engl J Med 356: 790-799. doi:10.1056/NEJMoa062607. PubMed: 17314338.17314338

[12] KingNJ, ParrEL, ParrMB (1998) Migration of lymphoid cells from vaginal epithelium to iliac lymph nodes in relation to vaginal infection by herpes simplex virus type 2. J Immunol 160(3): 1173‐1180. PubMed: 9570531.9570531

[13] GnannJW Jr, BartonNH, WhitleyRJ (1983) Acyclovir: Mechanism of action, pharmacokinetics, safety and clinical applications. Pharmacotherapy 3(5): 275-283. PubMed: 6359082.635908210.1002/j.1875-9114.1983.tb03274.x

The article "An Indole Alkaloid from a Tribal Folklore Inhibits Immediate Early Event in HSV-2 Infected Cells with Therapeutic Efficacy in Vaginally Infected Mice" was retracted in 2025. Reasons: errors in the methods; duplicated images; duplicated data; duplicate publication.

[14] KleymannG (2003) New antiviral drugs that target herpesvirus helicase primase enzymes. Herpes 10(2): 46-52. PubMed: 14577954.14577954

[15] StanberryLR (2004) Clinical trials of prophylactic and therapeutic herpes simplex virus vaccines. Herpes 11: 161A-169A. PubMed: 15319086.15319086

[16] MorfinF, ThouvenotD (2003) Herpes simplex virus resistance to antiviral drugs. J Clin Virol 26: 29-37. doi:10.1016/S1386-6532(02)00263-9. PubMed: 12589832. 12589832

[17] ReyesM, ShaikNS, GraberJM, NisenbaumR, WetherallNT et al. (2003) Task Force on Herpes Simplex Virus Resistance, Acyclovir-resistant genital herpes among persons attending sexually transmitted disease and human immunodeficiency virus clinics. Arch Intern Med 163(1): 76-80. doi:10.1001/archinte.163.1.76. PubMed: 12523920.12523920

[18] SwetterSM, HillEL, KernER, KoelleDM, PosavadCM et al. (1998) Chronic vulvar ulceration in an immunocompetent woman due to acyclovir- resistant, thymidine kinase-deficient herpes simplex virus. J Infect Dis 177(3): 543-550. doi:10.1086/514229. PubMed: 9498430. 9498430

[19] PosavadCM, KoelleDM, ShaughnessyMF, CoreyL (1997) Severe genital herpes infections in HIV-infected individuals with impaired herpes simplex virus-specific CD8^+^ cytotoxic T lymphocyte responses. Proc Natl Acad Sci U_S_A 94(19): 10289-10294. doi:10.1073/pnas.94.19.10289. PubMed: 9294203.9294203PMC23355

[20] ChatisPA, CrumpackerCS (1991) Analysis of the thymidine kinase gene from clinically isolated acyclovir-resistant herpes simplex viruses. Virology 180(2): 793-797. doi:10.1016/0042-6822(91)90093-Q. PubMed: 1846499.1846499

[21] DagarHS, DagarJC (1991) Plant folk medicines among Nicobarese of Katchal Island, India. Econ Bot 45: 114-119. doi:10.1007/BF02860056.

[22] ChattopadhyayD, DasS, MandalAB, ArunachalamG, BhattacharyaSK (2007) Evaluation of analgesic and antiinflammatory activity of *Ophiorrhiza* *nicobarica*, an ethnomedicine from Nicobar Islands, India. Oriental Pharm Experimental Med 7(4): 395-408. doi:10.3742/OPEM.2007.7.4.395.

[23] ChattopadhyayD, ArunachalamG, MandalAB, BhattacharyaSK (2006) Dose Dependent Therapeutic Antiinfectives from Ethnomedicines of Bay Islands. Chemother 52: 151-157. doi:10.1159/000092859.16636538

[24] BagP, ChattopadhyayD, MukherjeeH, OjhaD, MandalN et al. (2012) Antiherpes activities of bioactive fraction and isolated pure constituent of *Mallotus* *peltatus*: an ethnomedicine from Andaman Islands. Virol J:98. 10.1186/1743-422X-9-98PMC343055522624581

[25] ChiangLC, ChiangW, LiuMC, LinCC (2003) *In* *vitro* antiviral activities of *Caesapinia* *pulcherrima* and its related flavonoids. J Antimicro Chem 52: 194-198. doi:10.1093/jac/dkg291.12837746

The article "An Indole Alkaloid from a Tribal Folklore Inhibits Immediate Early Event in HSV-2 Infected Cells with Therapeutic Efficacy in Vaginally Infected Mice" was retracted in 2025. Reasons: errors in the methods; duplicated images; duplicated data; duplicate publication.

[26] VillamilSM, AlcheLE, CotoCE (1995) Inhibition of herpes simplex virus type-1 multiplication by meliacine a peptide of plant origin. Antivir Chem Chemother 6: 239-244.

[27] LinLT, ChenTY, ChungCY, NoyceRS, GrindleyTB et al. (2011) Hydrolyzable Tannins (Chebulagic Acid and Punicalagin) Target Viral Glycoprotein-Glycosaminoglycan Interactions to Inhibit Herpes Simplex Virus 1 Entry and Cell-to-Cell Spread. J Virol 85(9): 4386-4398. doi:10.1128/JVI.01492-10. PubMed: 21307190.21307190PMC3126266

[28] KanekiyoK, HayashiK, TakenakaH, LeeJB, HayashiT (2007) Anti-herpes simplex virus target of an acidic polysaccharide, nostoflan, from the edible blue-green alga *Nostoc* *flagelliforme* . Biol Pharm Bull, 30(8): 1573-1575. doi:10.1248/bpb.30.1573. PubMed: 17666824.17666824

[29] PiretJ, RoyS, GagnonM (2002) Comparative study of mechanism of herpes simplex virus in activation by sodium lauryl sulphate and n-lauroylsarcosine. Antimicrob Agents Chemother 46: 2933-2942. doi:10.1128/AAC.46.9.2933-2942.2002. PubMed: 12183250.12183250PMC127445

[30] FraziaSL, AmiciC, SantoroMG (2006) Antiviral activity of proteasome inhibitors in herpes simplex virus-1 infection: role of nuclear factor-κβ. Antiviral Therapy 11: 995-1004. PubMed: 17302369.17302369

[31] WangQY, ZhouC, JohnsonKE, ColgroveRC, CoenDM et al. (2005) Herpes viral latency-associated transcript gene promotes assembly of heterochromatin on viral lytic-gene promoters in latent infection. Proc Natl Acad Sci USA 102(44): 16055-16059. doi:10.1073/pnas.0505850102. PubMed: 16247011.16247011PMC1266038

[32] ZhouC, KnipeDM (2002) Association of Herpes Simplex Virus Type 1 ICP8 and ICP27 Proteins with Cellular RNA polymerase II Holoenzyme. J Virol 76(12): 5893-5904. doi:10.1128/JVI.76.12.5893-5904.2002. PubMed: 12021322.12021322PMC136207

[33] LiangY, VogelJL, NarayananA, PengH, KristieTM (2009) Inhibition of the histone demethylase LSD1 blocks α-herpesvirus lytic replication and reactivation from latency. Nat Med 15(11): 1312-1317. doi:10.1038/nm.2051. PubMed: 19855399.19855399PMC2783573

[34] ReedLJ, MuenchH (1938) A simple method of estimating fifty percent endpoints. Am J Hyg 27: 493-497.

[35] CocktonJR, WynnJB (1952) The use of surface active agents in pharmaceutical preparations: the evaluation of emulsifying power. J Pharm Pharmacol 4: 959-971. doi:10.1111/j.2042-7158.1952.tb13229.x. PubMed: 13000672.13000672

[36] GhoshS, SamantaA, MandalNB, BannerjeeS, ChattopadhyayD (2012) Evaluation of wound healing activity of methanolic extract of *Pedilanthus* *tithymaloides* (L.) Poit leaf and its isolated active constituents in topical formulation. J Ethnopharmacol 142(3): 714-722. doi:10.1016/j.jep.2012.05.048. PubMed: 22683906.22683906

The article "An Indole Alkaloid from a Tribal Folklore Inhibits Immediate Early Event in HSV-2 Infected Cells with Therapeutic Efficacy in Vaginally Infected Mice" was retracted in 2025. Reasons: errors in the methods; duplicated images; duplicated data; duplicate publication.

[37] KurokawaM, HozumiT, TsuritaM, KadotaS, NambaT et al. (2001) Biological Characterization of Eugeniin as an Anti-Herpes Simplex Virus Type 1 Compound *in* *Vitro* and *in* *Vivo* . J Pharmacol Exp Ther 297: 372-379. PubMed: 11259565.11259565

[38] BerrouguiH, Martín-CorderoC, KhalilA, HmamouchiM, EttaibA et al. (2006) Vasorelaxant effects of harmine and harmaline extracted from *Peganum* *harmala* L. seed's in isolated rat aorta. Pharmacol Res 54: 150-157. doi:10.1016/j.phrs.2006.04.001. PubMed: 16750635. 16750635

[39] WangX, GengY, WangD, ShiX, LiuJ (2008) Separation and purification of harmine and harmaline from *Peganum* *harmala* using pH-zone-refining counter-current chromatography. J Sep Sci 31: 3543-3547. doi:10.1002/jssc.200800322. PubMed: 18844206.18844206

[40] ZhengXY, ZhangZJ, ChouGX, WuT, ChengXM et al. (2009) Acetylcholinesterase inhibitive activity-guided isolation of two new alkaloids from seeds of *Peganum* *nigellastrum* Bunge by an *in* *vitro* TLC- bioautographic assay. Arch Pharm Res 32: 1245-1251. doi:10.1007/s12272-009-1910-x. PubMed: 19784581.19784581

[41] JahanianiF, EbrahimiSA, RahbarRN, MahmoudianM (2005) Xanthomicrol is the main cytotoxic component of *Dracocephalum* *kotschyii* and a potential anti-cancer agent. Phytochem 66: 1581-1592. doi:10.1016/j.phytochem.2005.04.035. PubMed: 15949825.15949825

[42] StanfordJA, FowlerSC (1998) At low doses, harmaline increases forelimb tremor in the rat. Neurosci Lett 241: 41-44. doi:10.1016/S0304-3940(97)00974-9. PubMed: 9502211.9502211

